# HMGB1 Upregulates RAGE to Trigger the Expression of Inflammatory Factors in the Lung Tissue in a Hypoxic Pulmonary Hypertension Rat Model

This article has been retracted.

**DOI:** 10.1155/2022/6823743

**Published:** 2022-07-19

**Authors:** Wen-Juan Li, Zhi-Peng Wen, Yan Xing, Jing-Ping Yang, Xi-Yuan Xu, Hong-Yan Wang, Wen-Yan Zhu, Yue-Hua Li

**Affiliations:** ^1^Departments of Respiratory & Critical Medicine, Inner Mongolia Baogang Hospital, Baotou, 014010 Inner Mongolia, China; ^2^Departments of Urology, Inner Mongolia Baogang Hospital, Baotou, 014010 Inner Mongolia, China

## Abstract

Hypoxic pulmonary hypertension (HPH), a form of pulmonary hypertension (PH) caused by hypoxia, could cause serious complications and has a high mortality rate, and no clinically effective treatments are currently available. In this study, we established an HPH preclinical model in rats by simulating clinicopathological indicators of the disease. Our results showed that high mobility group box-1 protein (HMGB1) aggravated the clinical symptoms of HPH. We aimed at establishing protocols and ideas for the clinical treatment of HPH by identifying downstream HMGB1 binding receptors. Our investigation showed that continuous hypoxia could cause significant lung injury in rats. ELISA and western blotting experiments revealed that HPH induces inflammation in the lung tissue and increases the expression of a hypoxia-inducible factor. Testing of lung tissue proteins *in vivo* and in human pulmonary artery endothelial cells *in vitro* revealed that the HMGB1-mediated increase in the receptor for advanced glycation end products (RAGE) expression promoted inflammation. In summary, we successfully established an HPH rat model providing a new model for preclinical HPH research and elucidated the role of HMGB1 in HPH. Furthermore, we describe that HMGB1 induced inflammation in the HPH model via RAGE, causing severe lung dysfunction. This study could potentially provide novel ideas and methods for the clinical treatment of HPH.

## 1. Introduction

Pulmonary hypertension (PH) is a physiological phenomenon that develops in the case of multiple lung diseases past a certain stage. Hypoxic PH (HPH), a form of PH caused by hypoxia, can lead to serious complications and has an extremely high mortality rate. HPH severely impacts the physical and mental health of patients, increasing their social and medical burden, as well as the risk of long-term disability [1, 2]. No specific HPH treatments are currently available, and most available HPH treatments cause systemic stress changes and have several side effects, making this an urgent clinical problem.

Our preliminary studies showed that the gene and protein expression of high mobility group box-1 (HMGB1) protein significantly increased in the lung tissue and serum samples of HPH model rats. The increase in HMGB1 promoted the expression of inflammatory factors in the lung tissue, thereby worsening HPH pathology. HMGB-1, a member of the HMG-box family, is an abundant and widely expressed protein that plays multiple roles in a variety of pathophysiological processes. HMGB1 is passively released from necrotic or damaged cells and might be actively secreted from immune cells or tissues under hypoxic conditions [3, 4]. HMGB-1 enters the extracellular space, binds to various receptors, and functions as a damage-associated molecule. HMGB-1 can also stimulate inflammatory signaling pathways such as the interferon (IFN) and nuclear factor kappa B (NF-*κ*B) pathways, induce the release of proinflammatory cytokines, and initiate an inflammatory response with accelerated circulation. Several studies have shown that HMGB-1 plays an important secondary role in HPH. This study is aimed at establishing *in vivo* and *in vitro* models of HPH to identify the downstream signaling targets of HMGB-1, thereby providing novel ideas for the clinical treatment of this disease.

## 2. Materials and Methods

### 2.1. Animals

Seven-to-eight-week-old male isogenic SD rats (Charles River, Beijing, China), weighing 140-160 g, were given standard rat chow and maintained in an environment with clean purified water. All animal experiments were approved by the Animal Ethical Committee of Medical University and were performed in accordance with the *Guide for the Care and Use of Laboratory Animals*.

### 2.2. HPH Model Establishment

SD rats were randomly divided into 3 groups based on their body weight: a normal (NC), an HPH, and an HPH-anti-HMGB1 group (10 rats per group). Animals in the HPH group were placed in an oxygen chamber, and a hypoxic model was established each day (air content adjusted to 10% oxygen, 85% nitrogen, and 5% carbon dioxide). The HPH+anti-HMGB1 group was injected intraperitoneally with 250 *μ*g/mouse recombinant anti-HMGB1 antibody (Abeam, USA) once every seven days during model establishment. Animals in the NC group were raised in normal air. All other conditions were the same in all three groups. The lung tissue sampling was performed 28 consecutive days after model establishment.

After model establishment, the animals were anesthetized with 20% ethyl carbamate; blood was then collected from the abdominal aorta, and the plasma was separated and stored in a -80°C freezer. The heart and lung tissues were carefully separated; the heart was dissected and the lung tissue was lavaged. The lavage process was as follows: the trachea was cut, and a tube was inserted; 15-20 mL normal saline was injected via the tube into the bronchus for alveolar lavage, and bronchoalveolar lavage fluid from six zones was drawn out and stored at 4°C. All lung tissue samples were collected and divided into two parts for storage. One part was fixed in 4% paraformaldehyde for hematoxylin and eosin (HE) staining, with the fixative covering the entire tissue. The other part was divided into two Eppendorf tubes and stored at -80°C for total RNA and protein extraction. The atria and great blood vessels of the heart were removed, and the left ventricle, ventricular septum, and right ventricle were isolated, weighed, and recorded. The right ventricular hypertrophy index was calculated using the formula RVHI = RV/(LV + S).

### 2.3. HE Staining

The lung tissues were immersed in 4% formalin paraformaldehyde. After dehydration with different concentrations of xylene, the lung tissues were embedded in paraffin. Lung tissue sections were stained with hematoxylin and eosin solutions for 10 min and 1 min, respectively. These sections were then microphotographed by a light microscope.

### 2.4. Detection of HMGB1, HIF-1, IL-1b, TLR4, and NF-*κ*B

The detection of HMGB-1, HIF-1, IL-1b, IL-6, TLR4, and NF-*κ*B in rat bronchoalveolar lavage fluid was performed according to the instructions of the enzyme-linked immunosorbent assay (ELISA) kits.

### 2.5. Western Blotting (WB)

The protein expression of HMGB-1 and RAGE in the lung tissue samples was investigated using WB. We loaded 30 *μ*g of sample per well and performed sodium dodecyl sulfate-polyacrylamide gel electrophoresis (SDS-PAGE) using a 10% Tris-glycine polyacrylamide gel. After electrophoresis, the proteins in the gel were transferred onto a polyvinylidene fluoride (PVDF) membrane. The membrane was blocked with 5% skim milk for 1 h at 37°C and incubated with the primary antibody overnight at 4°C. The membrane was rinsed four times (5 min each) with PBST and then incubated with anti-rabbit IgG (1 : 2000) secondary antibody for 90 min. An enhanced chemiluminescence (ECL) WB detection kit was used to detect immunolabeled protein bands. Densitometry was used to quantify protein levels. All experiments were performed independently in triplicates, and the average values were used for comparisons.

### 2.6. Effect of HMGB1 on the Expression of Inflammatory Factors in Human Pulmonary Artery Endothelial Cells (HPAECs)

HPAECs (ATCC American Type Culture Collection) in the growth phase were divided into four groups: a blank normoxia control, a hypoxia, a normoxia+HMGB1, and a hypoxia+anti-HMGB1 group. After the cells were passaged and adhered to the plate for 6 h, they were incubated under normoxic or hypoxic conditions and subjected to corresponding treatments (1 *μ*g/mL HMGB1 or 5 *μ*g/mL anti-HMGB1) depending on the group for 24 h. After treatment, the cell supernatant and cellular proteins were collected and used to detect the expression of IL-1*β* and IL-6 and of HMGB1 and RAGE, respectively.

### 2.7. Statistical Analysis

GraphPad Prism 7.0 analysis and graphing software and SPSS 21.0 software were used for the statistical analysis of the data. Data were expressed as the mean ± standard deviation (mean ± SD). The data were first tested for normality before analysis. Data conforming to the normal distribution were analyzed by one-way and multifactor analyses of variance. Differences with *p* < 0.05 were considered statistically significant.

## 3. Results

### 3.1. Successful Establishment of an HPH Rat Model

After 28 days in hypoxic conditions, the weights of rats in the HPH and HPH+anti-HMGB-1 group were lower than those of the animals in the NC group (*p* < 0.05). Clinical manifestations included delayed reaction time, partial loss of fur, impaired consciousness, and decreased activities. The weight of the rats in the HPH+anti-HMGB-1 group recovered compared with that of animals in the HPH group, and the difference was statistically significant (*p* < 0.05, Figure 1(a)).

Twenty-eight days after model establishment, the RVHI of both the HPH and HPH+anti-HMGB-1 groups was significantly higher than that of the NC group (Figure 1(b)). After the model establishment, the pulmonary arteries of each group were stained with HE. The observation of the tissue sections showed that the NC group had normal pulmonary artery wall structure, while the HPH group exhibited pulmonary artery wall thickening that caused severe narrowing of the lumen; the HPH+anti-HMGB-1 group also exhibited pulmonary artery wall thickening and narrowed lumen, but the narrowing was less severe than in the HPH group (Figure 1(c)). These results show that hypoxia can cause significant weight loss, right heart hypertrophy, and pulmonary artery tissue damage in rats, as well as PH. The injection of anti-HMGB-1 significantly ameliorated the damage to the pulmonary arteries in the hypertension model.

### 3.2. Inflammatory Factor Expression in the HPH Model Rat Alveoli

Compared to the NC group, the expression of HMGB-1, TLR4, IL-1*β*, IL-6, and HIF-1 in the bronchoalveolar lavage fluid of the HPH and HPH+anti-HMGB-1 groups significantly increased. Compared to the HPH group, the secretion of HMGB-1, TLR4, IL-1*β*, IL-6, and HIF-1 in the HPH+anti-HMGB-1 group significantly decreased (*p* < 0.05). These results indicate that the development of HPH can induce inflammation in the lung tissue, which has a significant association with HMGB1 expression. HIF is a hypoxia-inducible factor and plays an important role in hypoxia and its associated pathophysiological processes. In the HPH model, the expression of HIF-1 is significantly increased and is correlated with HMGB1 content.

### 3.3. HMGB1 and RAGE Expression in the Lung Tissue of HPH Model Rats

HMGB-1 and RAGE expression in the HPH group increased significantly compared with that in the NC group, indicating that HPH can promote HMGB1 and RAGE protein expression. The injection of HMGB1 significantly inhibited this expression of RAGE protein. RAGE is an important HMGB1 receptor and is abundant in the lung tissue, primarily expressed on the outer surface of the basal cell membrane of alveolar type II and alveolar type I epithelial cells. RAGE and HMGB1 expression and the secretion of inflammatory factors in the alveoli were increased in HPH model rats. The anti-HMGB1 supplementation reduced the RAGE protein expression and the secretion of inflammatory factors (Figures 2 and 3).

### 3.4. HMGB1 Protein Expression in HPAECs

HMGB1 protein expression in HPAECs was determined after different treatments. Hypoxia significantly promoted HMGB1 protein expression, and anti-HMGB1 significantly inhibited HMGB1 expression, indicating that anti-HMGB1 significantly antagonizes HMGB1 expression (Figure 4).

### 3.5. Inflammatory Factor IL-1*β* and IL-6 Content in HPAEC Supernatant

The expression of the inflammatory factors interleukin-1*β* (IL-1*β*) and IL-6 in the supernatant of HPAECs was determined after different treatments. The supernatant of the HPH cells and normal cells with HMGB1 added exacerbated inflammation, as evidenced by the increased secretion of IL-1*β* and IL-6 (Figure 5). The anti-HMGB-1 supplementation to the hypoxia model significantly reduced the production of the inflammatory factors IL-1*β* and IL-6, indicating that HMGB1 promotes inflammation.

### 3.6. RAGE Protein Expression in HPAECs

Determination of RAGE protein expression in cellular proteins showed that both hypoxia and HMGB1 increased RAGE expression, whereas anti-HMGB1 abrogated hypoxia-induced increase in RAGE protein expression (Figure 6). Exposure of HPAECs to hypoxia, anti-HMGB1 supplementation, and other treatments showed that both HMGB1 and hypoxia promoted the expression of the inflammatory factors IL-6 and IL-1*β*. The relationship between HMGB1 and RAGE in cellular proteins was found to be that HMGB1 is located upstream of RAGE. HPH model establishment promoted HMGB1 secretion, which in turn further activated RAGE and promoted inflammation.

## 4. Discussion

The precise HPH pathogenic mechanism is currently unknown but is primarily characterized by excessive pulmonary vasoconstriction and abnormal pulmonary vascular structure remodeling induced by hypoxia and leading to right heart failure. No clinically effective treatments are currently available for this disease, only symptomatic treatments, such as conventional oxygen inhalation, antibiotics, antiasthma treatments, improvement of cardiac function, and diuretics, which severely impact patient prognosis [5, 6]. Therefore, investigating the HPH pathogenic mechanism to provide new clinical treatment approaches should be a priority.

Studies have shown that HMGB-1 is a major regulator of HPH inflammation. Increased HMGB-1 levels not only reflect cellular damage but also induce multiple proinflammatory effects [7]. Studies have shown that the concentration of HMGB-1 in sputum and plasma samples of the patients with chronic obstructive pulmonary disease was significantly increased compared with that in a normal control group [8, 9], indicating that HMGB1 is involved in the remodeling of the airway and pulmonary vascular structure, which ultimately lead to HPH.

In the present study, we established an HPH rat model. The pathological histomorphology of the lungs was consistent with that of the HPH lung tissue. The differences in mean body weight and right heart hypertrophy index of the rats after 28 days were statistically significant among the three groups, suggesting the successful establishment of the HPH model. These results are consistent with those of previous studies. The expression of TLR4, IL-1*β*, and IL-6 in the bronchoalveolar lavage fluid, determined by ELISA, and HMGB1 and RAGE protein expression in the lung tissue, determined by WB, were both higher in the HPH group than in the control. These results indicate that the HMGB-1/TLR4/NF-*κ*B signaling pathway is activated during HPH, and the upregulated IL-1*β* and IL-6 are involved in the inflammatory response in HPH. HIF is an oxygen sensor. In a previous study, lentiviral transfection of HIF-1*α* into rat pulmonary blood vessels showed that the inhibition of HIF-1*α* expression in pulmonary blood vessels effectively alleviated chronic HPH and pulmonary vascular remodeling. The hypoxic stimulation did not cause HPH in mice with HIF-1*α* knocked out in pulmonary artery smooth muscle cells [10]. Studies have shown that HIF-1 participates in energy metabolism reactions. HIF-1*α* is strongly expressed under hypoxia and participates in glycolysis, which promotes the accumulation of lactic acid and leads to the formation of a slightly acidic environment [11, 12]. The present study showed significantly higher HIF-1 expression in the bronchoalveolar lavage fluid in the HPH group than in the NC group and in the HPH group than in the HPH+anti-HMGB-1 group and higher expression in the HPH+anti-HMGB-1 group than in the NC group. In summary, we conclude that HIF-1 expression is increased in the HMGB1-mediated HPH inflammatory response and plays an important role. Moreover, we confirmed that increased HIF-1 expression leads to lactic acid accumulation and the formation of a slightly acidic environment. These results are in good agreement with other related reports in the literature [13].

RAGE is an important receptor of HMGB1 and is abundant in the lung tissue, being primarily expressed on the outer surface of the basal cell membrane of alveolar type II and alveolar type I epithelial cells [14, 15]. The present study confirmed through both *in vivo* and *in vitro* experimental models that hypoxia and HMGB-1 significantly promote RAGE expression. When HMGB-1 is inhibited, RAGE protein levels are significantly downregulated, indicating that HMGB-1 and RAGE have an important relationship. RAGE directly activates the inflammasome signaling pathway in the cells [16], triggering inflammatory reactions and promoting the secretion of IL-1*β* and other inflammatory factors. Studies have found that inhibiting HMGB-1 effectively alleviates the symptoms of PH, which is consistent with the finding of the present study that HMGB1 plays a major role in PH. The inflammatory pathway in the lung tissue activated by RAGE through HMGB1 causes severe damage to the lung tissue and leads to severe lung dysfunction.

## 5. Conclusions

In this study, a rat model of HPH was successfully established, providing a new model for preclinical research on HPH, and the role of HMGB1 in HPH was elucidated. Furthermore, HMGB1 was found to induce inflammation in the model via RAGE, which causes severe lung dysfunction in HPH. However, only a single downstream effector of HMGB1 was investigated in the present study, and research on the pathogenic mechanism of HMGB1 in HPH is still lacking. More thorough studies are needed in the future to provide more avenues and methods for the clinical treatment of HPH.

## Figures and Tables

**Figure 1:** Changes of rats 28 days after model establishment: (a) body weight changes, (b) right ventricular hypertrophy, and (c) pathological section of pulmonary artery. ^∗^*p* < 0.05 compared to the NC group. ^#^*p* < 0.05 compared to the HPH group. *n* = 6. 100x magnification.

**Figure 2:** Detection of HMGB-1, TLR4, IL-1*β*, IL-6, and HIF-1 protein expression in rat bronchoalveolar lavage fluid by ELISA. ^∗^*p* < 0.05 compared to the NC group. ^#^*p* < 0.05 compared to the HPH group.

**Figure 3:** HMGB1 and RAGE protein expression in lung tissue of rats among different groups. All WB represent data from 3 independent repeats.

**Figure 4:** HMGB1 expression in HPAECs after different treatments. ^∗^*p* < 0.05 compared to the NC group. ^#^*p* < 0.05 compared to the HPH group.

**Figure 5:** IL-6 and IL-1*β* expression in HPAEC supernatant after different treatments. ^∗^*p* < 0.05 compared to the NC group. ^#^*p* < 0.05 compared to the HPH group.

**Figure 6:** Determination of RAGE expression in HPAEC proteins after different treatments. ^∗^*p* < 0.05 compared to the NC group. ^#^*p* < 0.05 compared to the HPH group.

## Data Availability

The data used and/or analyzed during the current study are available from the corresponding author on reasonable request.
